RETRACTED

# Correlates, comorbidities, and suicidal tendencies of problematic game use in a national wide sample of Korean adults

**DOI:** 10.1186/s13033-017-0143-5

**Published:** 2017-05-11

**Authors:** Subin Park, Hong Jin Jeon, Jung Woo Son, Haesoo Kim, Jin Pyo Hong

**Affiliations:** 1 Department of Research Planning, Mental Health Research Institute, National Center for Mental Health, Seoul, South Korea; 2 Department of Psychiatry, Samsung Medical Center, Sungkyunkwan University School of Medicine, 81 Irwon-ro Gangnam-gu, Seoul, 06351 Republic of Korea; 3 Department of Psychiatry, Chungbuk National University Hospital, Chungbuk National University School of Medicine, Cheongju, South Korea

**Keywords:** Problematic game use, Comorbidity, Suicide, Korea

## Abstract

**Background:**

This study aimed to investigate the prevalence, correlates, comorbidities, and suicidal tendencies of problematic game use in a nationally representative sample of Korean adults.

**Methods:**

Of the 6022 subjects who participated in the 2011 Korean Epidemiologic Catchment Area study and completed the Composite International Diagnostic Interview 2.1, 1397 game users were evaluated for problematic game use using 9-item DSM-5 proposed criteria for Internet gaming disorder. Respondents who responded “yes” to five or more of the nine DSM-5 criteria were considered as problematic game users and the reminders were considered as normal game users.

**Results:**

4.0% (56/1397) of game users were classified as a problematic game user. Problematic game users were more likely to be in younger age group and live in urban area compared with normal game user. Problematic game use was positively associated with several psychiatric disorders including nicotine use disorder, depressive disorder, and anxiety disorder, but not associated with alcohol use disorder and obsessive-compulsive disorder, after adjusting for age, sex, and residential area. Problematic game use was significantly and positively associated with suicide plans, after controlling for psychiatric disorders as well as socio-demographic factors.

**Conclusion:**

Problematic game use is relatively prevalent in Korean adult population and highly comorbid with other psychiatric disorders and suicidality. Therefore, preventive strategy for problematic game use is needed for game users who were more likely to be addicted such as young adults in urban area, and mental health screening and appropriate treatment are needed for individuals with problematic game use.

## Background

Internet gaming disorder, a repetitive use of Internet-based games that leads to significant impairment or distress, was contemplated in the Diagnostic and Statistical Manual of Mental Disorders-5 (DSM-5) published in 2013 as a condition for further study [1].

RETRACTED

The prevalence rates of problematic game use ranged from 0.5 to 9.9% with variation according to the study population and diagnostic instrument (for a review: [2]). Recently, Festl et al. [3] examined the prevalence rate of problematic game use in a large general population study and reported differences in prevalence rates among adolescents (7.6%), young adults (3.3%), and older adults (3.0%). Only a few studies used instruments based on the DSM-5 to estimate prevalence rates of problematic game use or game addiction. Rehbein et al. [4] found the 1.2% prevalence rate in a school-aged population in German, and Lemmens et al. [5] found the 5.4% prevalence rate in a Dutch sample of adolescents and young adults. More recently, Kim et al. [6] reported that 13.8% of Korean sample of adults with ages ranging from 20 to 49 years met DSM-5 criteria of Internet game disorder using Web-based survey.

With regard to psychiatric comorbidities, several studies have found higher rates of depressive symptoms [6–11], social incompetence [3, 5, 12, 13], and attention-deficit hyperactivity disorder [14, 15] among problematic game users compared to normal users. There have been only limited data on the association between problematic game use and substance abuse. Some studies reported no differences in prevalence of alcohol use disorder between problematic game users and usual users, but illicit drug use were more common in problematic game users [10, 16, 17]. Addictive behaviors were also linked to increased suicidal ideation and suicide attempt in previous studies [18, 19]. Several studies have found higher rates of suicidal ideation and suicide plan among excessive game users compared to normal users [12, 20, 21]. However, these population samples most often include adolescents or young adults.

In South Korea, where more than 98% of the households have access to the internet [22], internet or video games are considered to be a major recreational activity, and game addiction is becoming a serious social problem [23, 24]. Given the lack of information from large nationally representative studies of a general population sample on problematic game use, we investigated the prevalence, correlates, and psychiatric comorbidities of problematic game use in a nationwide sample of Korean adults aged 18–70 years.

## Methods

### Sample

Our data was driven from the Korean Epidemiologic Catchment Area (KECA) study conducted in 2011 [25], which used the Korean version of the Composite International Diagnostic Interview (K-CIDI) [26]. The KECA study has been performed per 5 years by the Ministry of Health and Welfare of South Korea since 2001 to measure the lifetime and 12-month prevalence and the association with sociodemographic, and comorbidities of major psychiatric disorders in the Diagnostic and Statistical Manual of Mental Disorders, Fourth Edition (DSM-IV) among Korean adults. The 2011 KECA study selected participants using a stratified, multi-stage, clustered sample design, based on a population census performed by community registry offices in 2010. After the study objective and procedures were fully informed, only the participants who provided informed consent enrolled in the study. Among 7650 subjects initially selected, 6022 participants completed the face-to-face interview by trained lay interviewers while 1628 refused (78.7% response rate) [25]. For these 6022 participants, game use was initially assessed with the following question (i.e. yes/no): “Have you ever Internet or video game in the past 1 year?” Participants who answered “yes” to this question (n = 1397) were assessed for problematic game use using the DSM-5 proposed criteria for Internet gaming disorder. Game users (n = 1397) were more likely to be male (69.9 vs. 43.9%), younger (33.18 ± 11.67 vs. 45.88 ± 14.23 years), unemployed (40.4 vs. 26.3%), and in higher educational (55.3 vs. 39.8%, high school or more) and economic (68.2 vs. 59.4%, family income >1000$) status, compared to non-users. There were no significant differences in residential area between game users and non-users (81.2 vs. 79.1%, urban residence). The 2011 KECA was approved by the institutional review board of the Seoul National University College of Medicine.

RETRACTED

### Measurement

#### Problematic game use

We used the DSM-5 proposed criteria for Internet gaming disorder [1] to evaluate problematic game use. Because we include video game and smart phone game as well as Internet game, the term ‘Internet game’ was replaced by ‘game’. Participants who responded “yes” to five or more of the criteria were considered as problematic game users and the remainders were classified as normal game users. Information on time spent for game use on weekdays and weekend and subjective magnitude of the problem related to game use using 5-Likert scale (ranged from a little to very much) were also collected.

#### Psychiatric disorders

Psychiatric disorders were diagnosed with a fully structured diagnostic tool, the CIDI [27] that is designed for psychiatric diagnoses based on the definitions and criteria of the DSM-IV [28]. The K-CIDI [26] was developed following World Health Organization (WHO) guidelines [29]. Kappa values of K-CIDI were as follows: the inter-rater reliability 0.86–1.00; test/retest reliability 0.42–0.89; validity of the K-CIDI 0.50–1.00.

RETRACTED

#### Suicidality

K-CIDI module on suicide were used to assess lifetime suicidality [26]. Lifetime suicidal ideation was assessed using the following dichotomous question (i.e. yes/no): “Have you ever seriously thought of committing suicide?” Lifetime suicide plan was assessed using the following dichotomous question (i.e. yes/no): “Have you ever concretely planned suicide?” Lifetime suicide attempts were assessed using the following dichotomous question (i.e. yes/no): “Have you ever attempted suicide?” [30].

#### Other variables

Information on socio-demographic status (i.e. sex, age, educational years, family income, and occupation) was obtained using self-reported questionnaires from the 2011 KECA study [31].

### Statistical analysis

Weighted values were calculated for each respondent to adjust the data to approximate the national population with respect to age and sex, according to the 2010 Korean National Statistical Office census [31]. All statistical analyses were conducted on the weighted data.

Pearson’s Chi square test was performed to compare sex, age group, economic status, occupational status, and residential area between problematic game users and normal game users. Independent t test was performed to compare time spent on Internet or game use and subjective magnitudes of the problem between problematic game users and normal game users. Multivariate logistic regression analyses were performed to calculate the odds ratios (ORs) and 95% confidence intervals (CIs) of lifetime psychiatric disorders, after adjusting for socio-demographic factors that were significantly different between groups. We also performed multivariate logistic regression analyses to calculate the ORs and 95% CIs of lifetime suicidality, after controlling for psychiatric disorders as well as socio-demographic factors. We used SPSS (version 21.0; SPSS Inc. Chicago, IL) to perform the aforementioned statistical analyses, and p value less than 0.05 was considered to be significant.

## Results

The estimated prevalence of problematic game use among game users was 4.0% (95% CI 2.0–3.0) (56/1397). In particular, 4.9% of younger adults aged from 18 to 39 years, and 1.6% of older adults aged from 40 years and older had problematic game use. Problematic game users spent longer time for gaming compared with normal users (p < 0.001) and perceived more problem related to their game use (p < 0.001). Addictive game users were more likely to be in younger age group and live in urban area (p = 0.008) compared with normal game users. There were no significant group differences in gender and educational and economic status (Table 1).

RETRACTED

**Table 1:** Characteristics of problematic game users and normal game users

	Normal game users (n = 1341)	Problematic game users (n = 56)	t	p
	Mean (SD)	Mean (SD)		
Time spent for internet use, weekdays (hours/day)	1.95 (1.97)	5.45 (5.30)	4.49	<0.001
Time spent for internet use, weekend (hours/day)	1.94 (2.44)	6.75 (5.32)	6.27	<0.001
Subjective magnitude of the problem (1–5)	1.67 (1.01)	3.31 (1.25)	9.70	<0.001

	%	%	X^2^	p
Age (years)			7.94	0.005
18–39	72.2	89.3		
40 or older	27.8	10.7		
Gender			0.001	0.971
Male	69.9	69.6		
Female	30.1	30.4		
Education			0.08	0.781
Less than high school	44.7	42.9		
High school or more	55.3	57.1		
Occupation			2.27	0.132
Employed	51.3	41.1		
Unemployed	48.7	58.9		
Residence			6.93	0.008
Urban	80.6	94.6		
Rural	19.4	5.4		
Family income			0.75	0.386
≤1000$	31.6	37.8		
>1000$	68.4	62.2		

74.1% of problematic game users had a lifetime history of mental disorder which fulfilled DSM-IV diagnostic criteria, compared to 37.4% of normal game users. Problematic game use was associated with nicotine use disorder (AOR 2.47, 95% CI 1.24–4.91), depressive disorders (AOR 4.13, 95% CI 2.12–8.36), and several types of anxiety disorder, including post-traumatic stress disorder (AOR 6.64, 95% CI 2.07–21.29), generalized anxiety disorder (AOR 4.87, 95% CI 2.63–9.02), and specific phobia (AOR 2.86, 95% CI 1.25–2.54) after adjusting for age, gender, and residential area. However, there was no significant association of problematic game use with alcohol use disorder and obsessive-compulsive disorder (Table 2). Moreover, problematic game use was significantly associated with lifetime suicidal plan (AOR 3.77, 95% CI 1.50–9.48) after controlling for comorbid psychiatric disorders as well as age, gender, and residential area. However, there was no significant association of problematic game use with suicidal ideation and suicide attempt (Table 3).

**Table 2:** Odds ratios for psychiatric disorders among problematic game users and controls

	Normal game users (n = 1341)	Problematic game users (n = 56)	AOR (95% CI)	p
	%	%		
Alcohol use disorder	22.1	25.9	1.43 (0.76–2.69)	0.265
Nicotine use disorder	10.9	21.4	2.47 (1.24–4.91)	0.010
Depressive disorder	6.6	23.2	4.13 (2.12–8.06)	<0.001
Any anxiety disorder	8.8	30.4	4.49 (2.42–8.36)	<0.001
Generalized anxiety disorder	1.9	10.7	6.26 (2.40–16.31)	<0.001
Specific phobia	5.2	14.5	2.86 (1.25–6.54)	0.013
Obsessive-compulsive disorder	0.7	1.8	2.00 (0.22–17.86)	0.534
Post-traumatic stress disorder	1.2	7.1	6.64 (2.07–21.29)	0.001
Any DSM-IV psychiatric disorder	37.4	74.1	4.87 (2.63–9.02)	<0.001

*AOR* adjusted for age, gender, and residential area

**Table 3:** Odds ratios for lifetime suicidality among problematic game users and controls

	Normal game users (n = 1341)	Problematic game users (n = 56)	AOR (95% CI)	p
	%	%		
Suicidal ideation	17.4	30.4	1.20 (0.59–2.42)	0.615
Suicidal plan	2.8	16.1	3.77 (1.50–9.48)	0.005
Suicide attempt	3.9	3.6	0.54 (0.12–2.43)	0.445

*AOR* Odds ratios adjusted for age, gender, residential area, and psychiatric disorders listed in Table 2

RETRACTED

## Discussion

The present study investigated the prevalence, associated factors, psychiatric comorbidities, and suicidality of problematic game use in a national representative sample of Korean adults. Our results confirmed prior findings that reported the association of problematic game use with several psychiatric disorders such as depressive and anxiety disorders in adolescent or younger adult population. We extended the findings of previous studies on problematic game use by using a nationwide sample involving younger adults to older adults and by applying DSM-5 criteria for Internet gaming disorder.

The prevalence of problematic game use in our data (4.0%) is much lower than 13.8% prevalence rate in adults aged between 20 and 49 years found in the study by Kim et al. [6], which also used five cut point out of nine DSM-5 criteria for Internet gaming disorder. It might be due to the different sampling populations of two studies. While our data used nationally representative sample, which included the general population of Korean adults, Kim et al. [6] collected their data via online survey, in which heavy Internet users are more likely to be recruited. Festl et al. [3] found the prevalence rates to be 3.0% for young adults (19–39 years) and 3.3% for older adults in a representative study in Germany, which is comparable to 4.0% prevalence rate of our data. However, given the different assessment instrument they applied (i.e. 7-item gaming addiction short scale; cut-off point of four or higher) [5], it may not be viable to directly compare the two results.

Compared to normal users, problematic game users were found to spend larger time in gaming and to perceive their gaming activity to be more problematic. Particularly, on the weekend, individuals with problematic game use used about 3.5 times longer hours than normal users. Consistent with prior findings [3, 7, 32], the problematic game users were more likely to be in their younger adulthoods than normal users, which might be attributed to the easier access to the technology of young adults. In addition, problematic game users were more likely to live in urban areas than normal users, suggesting that gaming culture might be more pervasive in major cities. As gambling behaviors were found to be largely affected by neighborhood accessibility to gambling opportunities [33], gaming behavior might also be affected by the widespread PC cafes or easier access to diverse game contents at metropolitan cities. A similar trend was found in users of novel psychoactive substances probably due to the more widespread opportunities to attend recreational settings such as discos and nightclubs, commonly located in urban areas [34].

RETRACTED

Our findings support the established associations of problematic game use with psychiatric disorders (for a review: [2]). In our data, 74.1% of those with problematic game use were found to have at least one diagnosis of psychiatric disorder. As found in prior studies [7, 35, 36], problematic game use was associated with increased prevalence of depressive disorder and anxiety disorder including generalized anxiety disorder, specific phobia, and post-traumatic stress disorder. It was also found that problematic game users had significantly higher prevalence of nicotine use disorder, but not alcohol use disorder. Similarly, several studies revealed that people with gaming disorder reported higher use of illicit drugs or smoking cigarettes, but not alcohol [10, 16]. Future studies are needed to investigate the differential association of problematic game use with diverse substance use and its underlying mechanism.

Problematic game use was not significantly associated with obsessive-compulsive disorder in our data, unlike the significant association between problematic Internet use and obsessive-compulsive disorder found in prior studies [37–39]. It is compatible with prior findings that obsessive-compulsive disorder symptoms were more closely related to addictive use of social media than that of video game [40]. It could be suggested that the association of OCD with problematic Internet use previously reported might be due to the association of OCD with a certain type of Internet use other than gaming. For instance, excessive use of social media, which takes a large part of addictive Internet use [41], was found to be related to the fear of missing out rewarding experiences other may have, accompanied by obsessive and compulsive checking behaviors [42]. In contrast, problematic game users might have different motivation or reward mechanism of their addictive behavior.

Moreover, 30.4% of problematic game users reported lifetime suicidal ideation, and especially, problematic game users had more than five times higher prevalence of suicide plan than normal game users, even after controlling for psychiatric disorders as well as socio-demographic factors. Prior findings also reported that excessive game playing was linked to increased suicidal ideation and suicide plan among adolescents [12, 20] and adults [21]. Although problematic game use was not significantly associated with suicide attempt in this study, given the fact that risk of future attempted suicide may persist for longer years among suicide ideators with plan than those without plan [43], the significant association with suicide plan suggests the chronic suicide risk of problematic game users. Therefore, people with problematic game use require clinical attention as a high suicide risk group and need extensive management for their mental difficulties.

RETRACTED

Given the association of problematic game use with depression and suicidal ideation, a measurement of anhedonia, a symptom of depression that is uniquely associated with suicidality [44], might be needed in future studies. Difficulty in experiencing pleasure could lead to the excessive use of games in an attempt to decrease anhedonia, as found in users of psychoactive substances [45]. In the previous study, trait anhedonia prospectively predicted a greater likelihood of addiction to online/offline video games in the emerging adult population [46].

The limitations of this study are as follows. First, this cross-sectional study cannot determine causality between variables due to the cross-sectional design. For instance, our data cannot answer how psychiatric comorbidities contribute to problematic game use, or conversely how addictive symptoms affect the progress of other psychiatric symptoms. Second, our data focused on Korean adult population, and thus adolescent population was not included in our data. Given problematic game use was found to be more prevalent and severe among adolescents (e.g., [32]), our results might not fully reflect the magnitude of game addiction problem in Korea. Third, this study focused on individual-level characteristics that affect problematic game use rather than community-level factors. Because community-level factors such as area-level deprivation may play an important role in determining adverse consequences of addictive behaviors [47], further researches considering these factors are needed to clarify the interactive effects of individual- and community-level factors on problematic game use. Finally, we used the DSM-5 proposed criteria for Internet gaming disorder, but did not use any validated scales, such as the Internet Gaming Disorder Scale [5] or the Game Addiction Scale [48]. Further exploration of the pathological dimension of game use is best accomplished by the use of a validated scale.

## Conclusion

Our results revealed that problematic game use is relatively prevalent in Korean adult population and highly comorbid with other psychiatric disorders and suicidality. Therefore, preventive strategy for problematic game use is needed for game users who were more likely to be addicted such as young adults lived in urban area. Also, mental health screening and appropriate treatment for both game addiction and comorbid psychiatric disorder are needed for individuals with problematic game use.

RETRACTED

## Abbreviations

DSM: Diagnostic and Statistical Manual of Mental Disorders
KECA: Korean Epidemiologic Catchment Area
K-CIDI: Korean version of the Composite International Diagnostic Interview
WHO: World Health Organization
OCD: obsessive compulsive disorder
